The article "Study of Intelligent Wireless Network Management in the Context of Artificial Intelligence for the Improvement of Chinese Language Mandarin Test Training Programmes" was retracted in 2023. Reasons: unreliable results or conclusions; concerns about the data; concerns about the peer review; concerns about the citations.

# Study of Intelligent Wireless Network Management in the Context of Artificial Intelligence for the Improvement of Chinese Language Mandarin Test Training Programmes

**DOI:** 10.1155/2022/4944114

**Published:** 2022-09-24

**Authors:** Xi Luo, Haiyan Chen

**Affiliations:** ^1^Open College, Jiangxi Open University, Nanchang, Jiangxi, China; ^2^Vocational College, Jiangxi Open University, Nanchang, Jiangxi, China

## Abstract

One of the most prominent ways of communication between people is through language, which plays a significant role in expressing thoughts. Different ways of expressing a language can be through speech, writing, signing, or gesture. Each country has their own traditional language and they are getting upgraded with technology in a complex environment. The country of China is termed as Chinese and they follow a dialect named Putonghua. Besides this Putonghua, the people follow different dialects, but this Putonghua is considered the official dialect. Also, the Putonghua Proficiency Test is to test the fluency of Chinese-speaking skills. In the traditional system, the test is conducted by the authorities manually. This process will be difficult when multiple people appear for the test, and in some circumstances, complex situations will arise. Hence, technological advancement can be leveraged to simplify the processes. In this research, Chinese language learning and the Putonghua Test were performed with the implementation of the Deep Learning (DL) model. This process involves the design of a DL model for mobile phones and training the model according to the application. Later, the concept is implemented through intelligent wireless network communication for learning and testing of the language. LIDA is implemented in this research work to train the system with DL. The main functionality of LIDA is template matching, which is required for testing the proficiency of the Chinese language by the candidate in PPT. When the new LIDA model is compared to the existing Vector Spaced Model (VSM), it is found that the LIDA achieves 98.67% of the test accuracy.

## 1. Introduction

For the self-organizing neural network to be deemed a success, it has been used in far too many different fields. Each layer's interlayer link between winning neurons has a substantial impact on the nanowire's structural and physical properties [1]. Measurements of biological activity were employed in this investigation [2]. Biosensors can be used to create artificial neural networks, self-organizing networks, and multilayer perceptrons for water quality monitoring and control [3]. If a computer-aided approach is utilised, microcalcification patterns can be spotted more quickly [4]. Breast cancer tumours can be classified and compared using neural networks with multilayer perceptrons and modular and self-organizing characteristics [5]. Data show that multilayer self-organizing networks have a stronger influence on detection than other networks [6]. The thermal capacity of a dual-tube nanofluid heat exchanger was studied using a back propagation artificial neural network with a multilayer perceptron structure back propagation artificial neural network (ANN) [7]. The results of this experiment reveal that data intake and heat transport are connected [8]. It is also possible to use the network to predict other variables, such as the heat transfer coefficient and the pressure loss [9]. A self-organizing neural network technique that accurately anticipates link weight and a high-precision self-organizing neural network can be used to successfully and realistically estimate aero engine thrust [10]. The multilayer perceptron classifier beat the prior probabilistic neural network classifiers [11]. A multilayer perceptron and a self-organizing feature map show that activated trash may be used to generate direct biopower in a laboratory (SOFM) [12]. Power density and removal rate were significantly affected by the volume of activated sludge, as well as pH and process temperature [13]. An artificial neural network was able to recognise and record actual heart sounds when trained with improved annealing [14]. Based on their findings, researchers used self-organizing maps and multilayer perceptrons to determine that entrepreneurs who engaged in public support programmes had an increased chance of surviving. Brain maps with self-organizing networks were proven to be quite beneficial in this study [15]. A wide range of disciplines can be predicted using neural networks and data mining approaches [16].

On the other hand, the use of this word in Chinese language studies is extremely rare. In this study on Chinese language features [17], data mining and a multilayer self-organizing neural network are used to improve predictions and results in this study. Chinese pop music has seen a surge in global recognition in recent years, with particular success in the United States. In recent years, tourists from all over the world have been flocking to China because of the country's rich cultural heritage and stunning natural beauty [18]. A detailed awareness of the current economic realities in China is required in order to successfully train a foreign student in the Chinese language and cultural traditions [19]. This needs an in-depth understanding of both ancient and modern artefacts, among other things. Another reason why Chinese has been termed “the most difficult language in the world to master” is the classification system established by the United Nations Educational, Scientific, and Cultural Organization (UNESCO). As a result, due to the large number of tones in Mandarin, it is one of the most difficult dialects for non-native speakers to master [20]. The pronunciation of the Cantonese dialect can be distinguished by as many as nine unique tones. Due to the fact that both Hong Kong and Macau utilise Cantonese as their major language of instruction, they have each built their own educational system that is tailored exclusively to the language of instruction. In general, nontonal language speakers will have difficulty learning Chinese's four tones unless they have been exposed to the language since childhood or are currently residing in a Chinese-speaking region of the world, which is rare. No one is exempt, not even those who speak in hushed tones, from this rule. Despite the fact that musicians from Hong Kong and Macau are routinely shown on television, their Mandarin is not considered standard. In the classroom, it is customary to communicate using the “subject-object-subject” approach to communication. It is vital for Chinese language teachers to employ language, text, and other object media to improve children's physical and mental development, and artificial intelligence (AI) can support them in this effort [21].

When teaching Chinese as a foreign language, teachers must deal with “diversity” on a variety of levels, including cultural, linguistic, and knowledge (Mandarin). The resources utilised in Chinese schools represent a diverse spectrum of cultural and linguistic variety. The presence of students from all over the world in a single classroom will have a substantial impact on the overall learning environment. Teachers can utilise artificial intelligence to collect data on their students' characteristics and then provide it to them in the form of data or text, which can assist them in discovering their students' strengths and weaknesses [22]. To put it another way, there is not any getting away from it. Chinese language teachers who are tasked with a variety of instructional duties can benefit from the use of artificial intelligence as an assistant to help them do these jobs more efficiently. Teachers still have a role to play when it comes to teaching a foreign language since they must gather and synthesise knowledge; artificial intelligence, on the other hand, is unable to make accurate decisions. In addition to the transfer of knowledge, teaching interaction entails the application of knowledge from pedagogy, the Chinese language, psychology, and social psychology [23]. This study focused on evaluating the performance of the Chinese language and putonghua test and training programme using AI.

## 2. Materials and Methods

The proposed methodology makes use of both wireless networks and artificial intelligence in the PPT. “Putonghua” is the Chinese language with a standard pronunciation that is currently used all over the world, according to China. The PPT, commonly known as the PSC, is a spoken fluency test in Standard Chinese (Mandarin) administered by the PRC Ministry of Education. It is a requirement to pass this test because it is part of the eligibility criterion for job positions in the government, education, and broadcasting fields. The test includes reading 100 monosyllabic words & 100 polysyllabic words for the pronunciation test. The vocabulary test, reading test, fluency test, and speaking on the given topic constitutes the rest of the test. Candidates who pass the test are awarded a Certificate of Putonghua Proficiency Level at one of three levels: 1, 2, or 3, with grades A and B. The eligibility for jobs with respect to the scores will be allocated.

Wireless network technology is an advanced technology that has simplified human tasks to a minute level. A wireless network is a computer network that allows users to connect their devices to the Internet via wireless data connections. The data are transferred from Node-to-Node with the help of wireless network systems. Every individual is connected to the network via wireless data connections in smart phones. This technology is integrated with AI technology to obtain improved results. Artificial intelligence is defined as the use of computers to accomplish tasks that would normally need human intelligence, such as speech recognition, decision-making, visual inspection, and translation is given in Figure 1. Artificial intelligence technology is divided into several sub-branches, including deep learning technology and machine learning technology. Deep learning is a type of machine learning algorithm that replicates the operations of the human brain. It is employed in artificial intelligence technology to carry out various tasks. Data is extracted using artificial neural networks. Multiple layers of artificial neural networks are used in Deep Learning. Deep learning techniques such as voice recognition and speech recognition are used for the test. The tests are conducted online with the assistance of artificial intelligence. Tests for more number of candidates are made easy with this proposed system thus improving the PPT.

The multiprocessor learning method will be incorporated into a DL- Logical Intelligent Detection Algorithm (LIDA), and the several module classification methods will be deployed within the framework. We will, in particular, discuss the data's building approach and also the associated optimization methods based using a semisupervised multiprocessor for Chinese language and Putonghua testing and training programme learning.

(1) $$\begin{array}{c} M_{1}{\left\|h\right\|}^{2}=\overset{s_{0}+T_{0}}{\underset{s_{0}}{\int }}{\left|V^{T}h\right|}^{2}nm\times \sum h_{2}{\left\|h\right\|}^{2},\omega_{s0}\geq \sum 0,s\in E^{k}\text{.} \end{array}$$

The growing complexity of data processing in Equation (1) develops considerably as *M* is the length of character *M*_1_‖*h*‖^2^the structures reach all the way through in this Chinese language possibility suggested that many. The parameters of the model|*V*^*T*^*h*|^2^*nm* × ∑*h*_2_‖*h*‖^2^, *ω*_*s*0_ ≥ ∑0, *s* ∈ *E*^*k*^ are practically hard to estimate on existing IT infrastructure specify the Equation (2). The presence or absence of *b*^*k*^(*s*) in a phrase is totally governed by the preceding phrase, which is the Chinese language framework.

(2) $$\begin{array}{c} b^{k}\left(s\right)=\sum h_{2}{\left\|h\right\|}^{2},\omega_{s0}\in \lim_{g⟶0}\frac{1}{g^{p}}\overset{k}{\underset{g=0}{\sum }}{\left(-1\right)}^{g}\left(\begin{array}{c} k\\ g \end{array}\right)\int b\left(s-kg\right)\text{.} \end{array}$$

The resemblance of a set of words before a paragraph is determined exclusively by*b*^*k*^(*s*)=(*ρ*^*i*^*x*/|*ρ*^*i*^*x*|+*d*) the two or more phrases preceding it, which is the Chinese language framework is given in the following equation:

(3) $$\begin{array}{c} b^{k}\left(s\right)=\int b\left(s-kg\right)\neq \left(\frac{\rho^{i}x}{\left|\rho^{i}x\right|+d}\right)+\sum {∁}_{\sigma }\left(x-x^{0}\right)=0\text{.} \end{array}$$

In equation (4), *g*_*i*_(*h*) denotes the student's language level that aims to illustrate the distinction between the cognitive stage of the learner and the level of difficulty in learning materials.

(4) $$\begin{array}{c} g_{i}\left(h\right)=\sum h_{2}{\left\|h\right\|}^{2},\omega_{s0}\in \frac{b_{i}s_{i}-\rho^{i}x}{\left|\rho^{i}x\right|+d}+\overset{k}{\underset{g=0}{\sum }}{\left(-1\right)}^{g}\left(\begin{array}{c} k\\ g \end{array}\right)\text{.} \end{array}$$

*R*_*i*_^*n*^(*s*) represents the learner's progress reflects the distinction between the aid the audience grasp contained within the learning resource but also the knowledge notes which learner wishes to gain. The smaller the gap, the more closely the expertise scores of the learning resource match *ρ*^*i*^*xR*_*ij*_^*n*^(*s*) the learner's experience notes. This following equation calculates the quality of student competence notes.

(5) $$\begin{array}{c} R_{i}^{n}\left(s\right)=\overset{k}{\underset{g=0}{\sum }}{\left(-1\right)}^{g}\left(\begin{array}{c} k\\ g \end{array}\right)\pm \underset{j\in g}{\sum }\rho^{i}xR_{ij}^{n}\left(s\right)\text{.} \end{array}$$

(*n*, *h*; *b*, *s*) -the formulation of the problem of expenditure also with educational resources indicates Equation (6) the general going to have to spend details amongst training resources.

(6) $$\begin{array}{c} {R_{i}^{n}\left|b\right|}^{0.7}=\left(n,h;b,s\right)+\int_{-\infty }^{+\infty }b\left(s\right)h\left(R-s\right)\sigma^{-jb\tau }bs\pm \int b\left(s-kg\right)\neq \left(\frac{\rho^{i}x}{\left|\rho^{i}x\right|+d}\right)\text{.} \end{array}$$

The objectives of the period of education *V*_*k*_(*n*) highlight the variations in learning time necessary to complete instructional resources *b*_*i*_*V*_*i*_(*n*)=*ω*^*T*^*V*(*n*), and learning time consumption is represented in the following equation:

(7) $$\begin{array}{c} V_{k}\left(n\right)=\underset{j\in g}{\sum }\rho^{i}xR_{ij}^{n}\left(s\right)\in \overset{k}{\underset{i=1}{\sum }}b_{i}V_{i}\left(n\right)+\sum M^{T}V\left(n\right)\text{.} \end{array}$$

Equation (8) is a workable description of the personalized learning journey optimization technique, represents the learner's overall optimal solution performance and *E*_*g*,*k*_ the learning path established by comments thread function such as through altering coefficients.

(8) $$\begin{array}{c} E_{g,k}=\lim_{g⟶0}\frac{1}{g^{p}}\overset{k}{\underset{g=0}{\sum }}{\left(-1\right)}^{g}\left(\begin{array}{c} k\\ g \end{array}\right)\int b\left(s-kg\right)b\left(s-kg\right)\neq \overset{M}{\underset{{∁}^{2}}{\sum }}\frac{{\left\|{\;E}_{g,k}\right\|}^{2}}{{∁}^{2}}+\left(\frac{\left({\;E}_{g,k}*M\right)}{{3∁}^{2}}\right)\text{.} \end{array}$$

The approach divides notification of a propagation direction of the particle in Chinese into three stages: frequency resistance, identification, and social behaviour. The (( *E*_*g*,*k*_*∗M*)/3∁^2^) stance notification of a material within creation that is decided by the position *T* and creates the generation needs with motion orientation, as described in the following equation:

(9) $$\begin{array}{c} K=\overset{M}{\underset{i=1}{\sum }}\left[{∁}^{i\left({\;E}_{g,k}*M\right)}-{∁}^{-\rho^{2}/\varepsilon }\right]\geq \frac{\overset{O}{\underset{i=1}{\sum }}M_{i}V}{\overset{O}{\underset{i=1}{\sum }}V_{i}}\text{.} \end{array}$$

The situation of the*Mh* ± *Mn* particle has been characterised from the perspective of 3∁^2^ possibilities. In subspace, each particle's *M*_*i*_ ∈ *V* bit value is 0 or 1, and the equation is exactly as specified in Equations (10) (11).

(10) $$\begin{array}{c} Mh\pm Mn=\frac{\overset{O}{\underset{i=1}{\sum }}M_{i}V_{i}}{T}\left(M_{i}\in V\right)+\overset{k}{\underset{i=1}{\sum }}\left[s_{i}-\overset{i}{\underset{j=1}{\sum }}\left(n+\overset{\rho }{\underset{j=1}{\sum }}n_{ij}\beta_{j}\right)\geq 1+\overset{j}{\underset{i=1}{\sum }}\left(+\overset{s}{\underset{j=1}{\sum }}n_{ij}\beta_{j}\right)\right]=0\text{.} \end{array}$$

(11) $$\begin{array}{c} T_{j}=\frac{\left(\left({\;E}_{g,k}*M\right)/{3∁}^{2}\right)}{\left(1+\overset{4}{\underset{j=1}{\sum }}d_{j}h_{j}\right)}+\overset{i}{\underset{j=1}{\sum }}\left(n+\overset{\rho }{\underset{j=1}{\sum }}n\beta_{j}\right)\text{.} \end{array}$$

Similarly, only this kind of difficulty relationship in Equation (12) can be limited to such situations.

(12) $$\begin{array}{c} T_{5}=\overset{i}{\underset{j=1}{\sum }}\left(n+\overset{\rho }{\underset{j=1}{\sum }}n_{ij}\beta_{j}\right)\geq \overset{s}{\underset{j=1}{\sum }}\left(1+k_{5}h_{5}\right)+\underset{j\in g}{\sum }\rho^{i}xR_{ij}^{n}\text{.} \end{array}$$

That higher the *T*_5_ science test standard when *k*_5_*h*_5_, the optimum option is selected that also satisfies all of the restrictions.

The evaluation problem is broken into four categories: difficult problems (*k*  < 0.5), unlucky conditions (*k*  < 0.8), middle discussions (0.5 ≤ *k* ≤ 0.8), and easy replies (0.7 ≤ *k* ≤ 1). The standard language exam problem is structured as in the following equation:

(13) $$\begin{array}{c} MK=\overset{\rho }{\underset{i=1}{\sum }}\overset{i}{\underset{j=1}{\sum }}\left(n+\overset{\rho }{\underset{j=1}{\sum }}n_{ij}\beta_{j}\right)\geq 1+\overset{j}{\underset{i=1}{\sum }}\left.\left(n\right)+\overset{s}{\underset{j=1}{\sum }}n_{ij}\beta_{j}\right)\overset{\rho }{\underset{i=1}{\sum }}M_{i}k_{i}/\overset{\rho }{\underset{i=1}{\sum }}M_{i}\text{,} \end{array}$$

where *MK* is the ordinary difficulty of such a test; *M* denotes the set of questions on the Chinese language exam; *i* denotes the number of exam questions, *i*=0, 1,…*ρ*; *M*_*i*_ denotes the difficulties of an *i* test; and *M*_*i*_ denotes the *i* test score. Following Equations (14) and (15), several analytical methods were employed to obtain the evaluation region score frequency.

(14) $$\begin{array}{c} MK=\overset{\rho }{\underset{i=1}{\sum }}\rho^{i}xR_{ij}^{n}\left(s\right)\overset{\rho }{\underset{i=1}{\sum }}M_{i}k_{i}+\overset{s}{\underset{j=1}{\sum }}\left(1+k_{5}h_{5}\right)\text{,} \end{array}$$

(15) $$\begin{array}{c} M=\sum M^{T}V\left(n\right)+\overset{g}{\underset{h=1}{\sum }}\frac{\left(T_{h}-T_{O}\right)}{\sum_{j\in g}\rho^{i}xR_{ij}^{n}\left(s\right)}\text{.} \end{array}$$

Each objective test yields the same conditional probability of occurrence or nonoccurrence. These experiments is known as a huge Conditional probability scientific experiment is demonstrated in Equations (16) and (17).

(16) $$\begin{array}{c} M_{g}\left(g\right)=\overset{k}{\underset{i=1}{\sum }}b_{i}V_{i}\left(n\right)+\sum M^{T}V\left(n\right)\overset{h}{\underset{g=0}{\sum }}\left(\begin{array}{c} g\\ h \end{array}\right)M^{g}f^{g-h}\text{,} \end{array}$$

(17) $$\begin{array}{c} \int h=g^{M}<M=\overset{g}{\underset{h=1}{\sum }}\frac{\left(T_{h}-T_{O}\right)}{g}\text{.} \end{array}$$

## 3. Results and Discussion

The measures utilised to evaluate student performance for the language study are reliability, feasibility, efficiency, text mining quality, but also maximum retracement ratio, as shown in Figure 2.

Purity, recall rate, and difference in evaluation classes were the evaluation criteria used. The numerical representation of this Figure 2 is shown in Table 1.

Figure 3 displays the training and testing assessment processes, which have been analyzed and presented in chart style. In comparison to the existing system, the traditional test has demonstrated the least values of 50% greater than the traditional language and the recall rate of the procedures. The recall rate is higher in traditional language testing and training, and Chinese language and Putonghua. The valued representation of the discrepancies is shown in Table 2. The time it takes for data to travel from the teacher's node to the student's node is recorded. For the analysis, the WebKB8275 Chinese Language Dataset was employed.

Figure 4 depicts an online test-based performance analysis for the Chinese language. This online test employs the technologies WSN and DL methods. The analysis based on the traditional language test and train, online test, frequency, and recall rate is depicted in this graph. These parameters demonstrate performance swings ranging from 80% to 95%, as shown in Table 3.

Figure 5 displays a study of various online test prediction performed on students following training sessions. It is expected in this Putonghua test and other online tests that online tests are implemented with the concept of a smart or intelligent evaluation mechanism. The questions in this system are created automatically, and the results are evaluated automatically.

Table 4 compares the new Logical Intelligent Detection Method to the existing Fuzzy cohesion algorithm in terms of performance. The performance is evaluated in order to forecast the outcome of the test using various approaches.

According to the predicted test results, the proposed system has gained 2.87%, 2.42%, 1.11%, and 2.37% in contrast to the proposed model. While taking online lessons, wireless internetworking devices are used with the help of WSN and DL. The proposed system exhibits a consistent increase in performance across all metrics.  Figure 6 depicts a graphical representation of the discussed.

## 4. Conclusions

Since its inception, artificial intelligence (AI) has been widely adopted for human benefit across a wide range of fields. China's Ministry of Education and the Institute of Applied Linguistics (IAL) administer the Putonghua Proficiency Test (PPT), also known as Putonghua Shuiping Ceshi (PSC), a test of spoken fluency in Standard Chinese (Mandarin) (PRC). Aspirants must pass these tests since they are required for government, education, and broadcasting positions. A total of three grades and six levels comprise the PPT. It is customary for authorised faculty to administer this test by hand. The manual test results show a wide range of variations. In addition, the cost of conducting a test for a large number of candidates is prohibitive. As a result, an evaluation model with artificial intelligence is required to evaluate the testing procedure. Researchers will examine how intelligent wireless network management may help improve the Chinese language and the Putonghua examination and training programme in the context of artificial intelligence. The PPT uses wireless network technology and artificial intelligence to improve the testing and training procedures, and the ultimate goal is to improve the Chinese language using this way. The PPT made use of wireless network technology that included artificial intelligence and discovered it to be quite effective. The proposed model has provided an accuracy of 98%.

## Figures and Tables

**Figure 1:** Intelligent system for improvement in putonghua test.

**Figure 2:** Evaluation of specific performance to the improvement of Chinese language and putonghua test and training programme.

**Figure 3:** WebKB8275 Chinese language dataset test and training programme class time.

**Figure 4:** Online questionnaire Chinese language performance evaluation using WSN and AI techniques.

**Figure 5:** A performance comparison of exam date prediction in Chinese using WSN and DL techniques.

**Figure 6:** Analysis of online test prediction in Chinese language using existing WSN with deep learning.

**Table 1:** Evaluation of the testing and training program result analysis.

Program for testing and training	Purity	Recall rate	Difference between evaluation classes
Text mining effectiveness		14	13
Text mining's viability	30	15	15
Text mining reliability	25	19	25
Ration of maximum retracement	15	23	19
Quality of text mining	32	12	20

**Table 2:** Class time result analysis for the WebKB8275 Chinese language dataset.

Dataset WebKB8275 Chinese language	Training rate	Testing rate	Time based frequency (s)	Accuracy (%)
Vector space model (traditional)	175	300	0.89	85
Language: Chinese	101	245	0.98	91
Rate of recall	125	267	0.91s	92

**Table 3:** Analysis of online test results for the Chinese language using WSN and AI techniques.

Online exam	Frequency of the network	Analyzing test results	Algorithm for logical intelligent detection	Accuracy (%)
Traditional language assessment and training	89	92	95	93
Online exam	86	89	97	95
Frequency	93	84	98	92
Rate of recall	89	94	97	98

**Table 4:** Result analysis for online test prediction in Chinese language compared to existing system.

Algorithm	Questioner online based overall test prediction	Online Chinese language class based mining test	Online network frequency (WSN with DL)	Accuracy (%)
Logical intelligent detection algorithm (LIDA)	97.54	93.76	95.23	98.67
Existing method: vector space model (traditional)	94.67	91.34	94.12	96.32

## Data Availability

The data used to support the findings of this study are available from the corresponding author upon request.

## References

[1] Han J. (2017). Chinese language and duiwai hanyu jiaoxue (teaching Chinese as a foreign language). *Post-lingual Chinese Language Learning*.

[2] Kang Y. J. (2010). Significance of Chinese Classificatory Glossaries Teaching through the Translation Booksin the Joseon Dynasty. *Chinese Language Education And Research*.

[3] Aulestia V. H. (2019). The impact on a foreign langauge curriculum of foreign langauge television signals received from geosynchronous earth satellites. *IALL Journal of Language Learning Technologies*.

[4] Cool J. (2020). Intelligent wood machining monitoring using vibration signals combined with self-organizing maps for automatic feature selection. *International Journal of Advanced Manufacturing Technology*.

[5] Liu Q., Li H., Zhang Y., Zhao Z. (2019). Pattern recognition of messily grown nanowire morphologies applying multi-layer connected self-organized feature maps. *Journal of Materials Science & Technology*.

[6] Chen M., Yang Z., Liu W. J. Deep neural networks for Mandarin tone recognition.

[7] Shen P., Lu X., Li S., Kawai H. Conditional generative adversarial nets classifier for spoken language identification.

[8] Revay S., Teschke M. (2019). Multi-class language identification using deep learning on spectral images of audio signals. https://arxiv.org/abs/1905.04348.

[9] Masud M., Muhammad G., Alshamrani H., Cheikhrouhou O., Ibrahim S., Hossain M. S. (2020). Deep learning-based intelligent face recognition in IoT-cloud environment. *Computer Communications*.

[10] Dey P., Pal T. (2017). On improving generalization of classifiers using feature extraction. *International Journal of Control Theory and Applications*.

[11] Kumar S., Kumar V. (2019). Transfer learning in 2.5D face image for occlusion presence and gender classification. *Handbook of Research on Deep Learning Innovations and Trends*.

[12] Singh M., Singh D. (2021). Multi-modality medical image fusion technique using multi-objective differential evolution based deep neural networks. *Journal of Ambient Intelligence and Humanized Computing*.

[13] Hassan H., Aue A., Chen C. (2018). Achieving Human Parity on Automatic Chinese to English News Translation. https://arxiv.org/abs/1803.05567.

[14] Verma M., Buduru A. B. Fine-grained language identification with multilingual CapsNet model.

[15] Rezaei-Ravari M., Eftekhari M., Saberi-Movahed F. (2021). Regularizing extreme learning machine by dual locally linear embedding manifold learning for training multi-label neural network classifiers. *Engineering Applications of Artificial Intelligence*.

[16] Yang J., Wu S., Zhang D., Li Z., Zhou M. Improved neural machine translation with Chinese phonologic features.

[17] Wetzstein G., Ozcan A., Fan S. (2020). Inference in artificial intelligence with deep optics and photonics. *Nature*.

[18] Nishant R., Kennedy M., Corbett J. (2020). Artificial intelligence for sustainability: challenges, opportunities, and a research agenda. *International Journal of Information Management*.

[19] Jiménez-Luna J., Grisoni F., Schneider G. (2020). Drug discovery with explainable artificial intelligence. *Nature Machine Intelligence*.

[20] Lin X., Liu J., Zhang J., Lim S. J. (2020). A novel beam search to improve neural machine translation for English-Chinese. *Computers, Materials & Continua*.

[21] Shneiderman B. (2020). Human-centered artificial intelligence: reliable, safe & trustworthy. *International Journal of Human-Computer Interaction*.

[22] Qu X., Yang L., Ma K. (2021). A survey on the development of self-organizing maps for unsupervised intrusion detection. *Mobile Networks and Applications*.

[23] Wu S., Wang X., Wang L. Tencent neural machine translation systems for the WMT20 news translation task.

